# High Expression of PDE8B and DUOX2 Associated with Ability of Metastasis in Thyroid Carcinoma

This article has been retracted.

**DOI:** 10.1155/2021/2362195

**Published:** 2021-12-20

**Authors:** Zhenguo Sun, Xiaoshuai Yuan, Peng Du, Peng Chen

**Affiliations:** Department of Nuclear Medicine, The First People's Hospital of Lianyungang, The First Affiliated Hospital of Kangda College of Nanjing Medical University, Lianyungang City 222000, China

## Abstract

**Background:**

Hormone is an independent factor that induces differentiation of thyroid cancer (TC) cells. The thyroid-stimulating hormone (TSH) could promote the progression and invasion in TC cells. However, few genes related to hormone changes are studied in poorly differentiated metastatic TC. This study is aimed at constructing a gene set's coexpression correlation network and verifying the changes of some hub genes involved in regulating hormone levels.

**Methods:**

Microarray datasets of TC samples were obtained from public Gene Expression Omnibus (GEO) databases. R software and bioinformatics packages were utilized to identify the differentially expressed genes (DEGs), important gene module eigengenes, and hub genes. Subsequently, the Gene Ontology (GO) enrichment analysis was constructed to explore important biological processes that are associated with the mechanism of poorly differentiated TC. Finally, some hub gene expressions were validated through real-time PCR and immunoblotting.

**Results:**

Gene chip with category number GSE76039 was analyzed, and 1190 DEGs were screened with criteria of *P* < 0.05 and ∣log_2_foldchange | >2. Our analysis showed that human dual oxidase 2 (DUOX2) and phosphodiesterase 8B (PDE8B) are the two important hub genes in a coexpression network. In addition, the validated experimental results showed that the expression levels of both DUOX2 and PDE8B were elevated in poorly differentiated metastatic TC tissues.

**Conclusion:**

This study identified and validated that DUOX2 and PDE8B were significantly associated with the metastasis ability of thyroid carcinoma.

## 1. Introduction

Thyroid cancer (TC) is the most common endocrine malignancy in thyroid tissues, which is considered to be related to hormone levels and genetic predisposition factors [1]. Due to the characteristics of abnormal cell proliferation and the possibility of spreading to other parts of the body, the incidence of TC has increased rapidly in recent decades. According to the surveillance of National Cancer Institute, the epidemiology survey indicated that TC patients accounted for 3.4% of all annual diagnoses [2]. As of 2015, 3.2 million people worldwide suffered from TC [3].

In differentiated thyroid cancer, about 4% of patients have distant metastasis at diagnosis, while another 7% to 23% of patients develop metastatic disease within five years [4]. The lymph nodes, lungs, bones, and brain are common metastatic sites for TC cancer cells [5]. Studies have shown that the prognosis of patients with lung metastasis is poor [6]. Metastatic TC is more malignant and no effective treatment available currently [7]. Therefore, it is very important and urgent to reveal the molecular mechanism of TC metastasis which is very important and urgent. Previous studies have compared the gene expression profiles of TC tissues through microarray technology [8], RT-qPCR, and next-generation sequencing [9]. The differentially expressed mRNAs in TC have been reported in multiple reports. However, the identified differentially expressed mRNAs from different studies varied widely, and the critical expressed genes of metastatic TC still need to be further supplemented. Therefore, in this study, we collected TC-related gene microarray data profiles form Gene Expression Omnibus (GEO) and identified several metastasis-related genes and evaluated the gene expression levels in TC samples.

## 2. Materials and Methods

### 2.1. Microarray Data and Specimens

The gene mRNA microarray expression dataset of TC was downloaded from the Gene Expression Omnibus databases (GEO) [10], which was served as a public repository for gene expression datasets. Gene chip GSE76039 generated from GPL570 platform (Affymetrix Human Genome U133 Plus 2.0 Array) [11], including 20 anaplastic TC (ATC) and 17 poorly differentiated metastatic TC (PDMTC) samples. To obtain the relative gene expression levels in each sample, this dataset was normalized using quantile RMA normalization.

To validate the protein concentration of target genes, 10 paired thyroid cancer and adjacent noncancerous tissues were collected from patients with TC in Affiliated Hospital of Beihua University. The written informed consent was obtained from each patient. This protocol used in this study was approved by the Institutional Review Board of the Affiliated Hospital of Beihua University.

### 2.2. Identifying Differentially Expressed Genes

Significance of differentially expressed genes (DEGs) was screened by DEseq2 (version 1.30) package in R software (version 3.4.2) [12] according to the methods described previously [13]. Fisher's exact test was used to calculate the *P* value of null hypothesis. All genes were considered to be significantly differentially expressed with criteria of *P* < 0.05 and ∣log_2_foldchange | >2 (∣logFC | >2).

### 2.3. Weighted Gene Coexpression Network and Gene Modules

The weighted gene coexpression network based on the DEGs was constructed using WGCNA package in R software. Topological overlap matrix (TOM) was constructed after a weighted adjacency matrix established with a power value beta = 10 [14]. In the TOM object, the interconnectedness of two genes was assessed by the degree of their shared neighbors across the global network [15].

Each gene module represents a cluster of genes that have high topological overlap. All the gene modules were detected by averaging the stratified clustering of each group. The connectivity within gene modules was calculated using the in-module connection function in WGCNA package. The module eigengene (ME), as the first principal component, was used to evaluate the membership of a given gene module and the importance of genes in the network [16].

### 2.4. Enrichment Analysis of Differentially Expressed Genes

R software packages and bioinformatics tools were used to perform an enrichment analysis of the DEGs in biological process. The DEGs (mean logFC: 2.93) within the enrichment analysis results were mapped to Gene Ontology (GO) and Kyoto Encyclopedia of Genes and Genomes (KEGG) databases [17] through clusterProfiler [18] package. In the GO enrichment analysis, only the biological process category was considered. Significant DEGs were further examined using the gene set enrichment analysis (GSEA) to filter out up- or downregulated genes [19]. The DEGs list was preranked according to their logFC values produced in the gene expression association test. GSEA was performed on both all probes and subsets of the WGCNA modules with a similar concept of the GO and KEGG analyses.

### 2.5. Real-Time PCR

Total RNA was isolated from approximately 20 mg of tissue by TRIzol reagent (Invitrogen, USA) according to the instructions. Subsequently, 1 *μ*g of total RNA was subjected to cDNA synthesis using RevertAid RT Reverse Transcription (Invitrogen, USA). The primer sequences of PDE8B (F: 5′-AGTCAGCCCTTGAATGCTTTC-3′; R: 5′-GCATCGAAGTTCTGAGTTTGTCT-3′), DUOX2 (F: 5′-CTGGGTCCATCGGGCAATC-3′; R: 5′-GTCGGCGTAATTGGCTGGTA-3′), and GAPDH (F: 5′-GGAGCGAGATCCCTCCAAAAT-3′; 5′-GGCTGTTGTCATACTTCTCATGG-3′) were obtained from PrimerBank (https://pga.mgh.harvard.edu/primerbank) and synthesized from Invitrogen (Shanghai, China). The real-time PCR was performed by Fast SYBR™ Green Master Mix (Invitrogen, USA) on an ABI 7500 Real-time PCR system (ABI, USA) according to the manufacturer's instructions.

### 2.6. Immunoblotting

Total proteins were extracted from tissues using RIPA buffer containing proteinase inhibitors. Protein concentrations were measured using BCA kit (Invitrogen, USA). Approximately 50 *μ*g of each protein was loaded onto an SDS-PAGE gel. After electrophoresis, the proteins were transferred to the PVDF membrane. The PVDF membrane was incubated with the diluted primary antibodies overnight at 4°C (PDE8B, 1 : 500, CST; DUOX2, 1 : 500, CST; and GAPDH, 1 : 1000, CST). Subsequently, the membrane was incubated with anti-mouse IgG, HRP-linked antibody (1 : 1000, CST, USA). Finally, the enhanced chemiluminescence detection system (FluorChem, NatureGene Corp.) was used to detect the protein expression on the PVDF membrane.

### 2.7. Statistical Analysis

All data were processed and analyzed by IBM SPSS 24.0 software (Chicago, IL, USA). Student's *t*-test was used to evaluate the statistical differences and *P* < 0.05 was considered significant.

## 3. Results

### 3.1. Weighted Gene Coexpression Network of the DEGs

Differences in normalized expression data were analyzed after preprocessing (Figure 1). A total number of 1190 including 479 upregulated and 711 downregulated genes met the significant criteria (*P* < 0.05 and ∣logFC | >2) were screened (Figure 2(a)). Subsequently, weighted gene coexpression network of the 1190 DEGs was constructed by WGCNA package. Combined with the TOM, the hierarchical average linkage clustering method was applied to detect gene modules in the network. The gene modules are identified by the principle of dynamic tree cutting (deep split = 2, cut height = 0.99). In both the ATC and PDMTC groups, four gene modules were identified (Figure 2(c)). Genes which did not belong to any modules were ignored in this study and classified as grey module.

As expected, there was a high degree of correlation between gene modules. With the mean module membership or mean correlation of gene expression within the module eigengenes, the values of correlation coefficient vary from 0.65 to 0.91 across all gene modules (Figure 2(d)). A correlation test of module eigengenes was conducted and summarized in Figure 2(d), and all modules were significant after controlling the false discovery rate (FDR).

### 3.2. Biological Process Results of DEGs

GSEA was carried out with the DEGs except grey module through enrichment analysis, and the results met significant level *P* < 0.05 are listed in Table 1. The most important GO terminologies are mainly focused on thyroid gland development and hormone metabolic process (Figure 2(b), Table 1). In addition, all these GO terminologies were activated in PDMTC compared with the primary ATC samples, and most of the genes were upregulated (Figure 2(b)).

### 3.3. DEGs' Interaction in the Network

Hub genes with high degree represent critical roles in the regulation of TC status due to the important biological significance in the whole network. To identify hub genes in top significant GO terminologies, the in-module connectivity was calculated with the signed TOM based on an adjacency matrix. The top strongest connections of genes within the modules were extracted with a threshold value of 0.25. The results showed that DUOX2 and PDE8B were the two core genes with highest connectivity (Figure 3(a)). Due to the same genes in different biological processes, the overlap between the processes was inevitable and the screened genes may be involved in multiple processes. Therefore, constructing a network of interactions of main biological processes was necessary for exploring the signal transmission in pathway. The biological processes in the coexpression network that primarily associated with the thyroid and hormonal metabolic processes are almost significantly enriched (Figure 3(b)).

### 3.4. Expressions of PDE8B and DUOX2

To confirm the gene expression levels of DUOX2 and PDE8B in thyroid cancer tissues, the mRNA levels of PDE8B and DUOX2 in human TC and adjacent noncutaneous tissues were detected by real-time PCR. The results showed that both PDE8B and DUOX2 were significantly increased in all TC tissues compared with adjacent noncutaneous tissues (Figure 4(a)). To further evaluate expression levels of two proteins, immunoblot experiment was performed according to the instructions and the results showed that the protein levels of PDE8B and DUOX2 were also elevated in TC samples (Figure 4(b)).

## 4. Discussion

PDMTC normally behave more aggressively and are associated with worse survival rates than well-differentiated patients [20]. Therefore, it is necessary to exploit novel candidate genes to develop targeted therapies [21]. In this study, we aimed to investigate the gene expression characteristics of TC patients to promote better understand the mechanism of PDMTC metastasis.

WGCNA has been widely used for data mining, especially in studying biological networks and analyzing gene expression data to find intramodular hub genes [22]. Through WGCNA and enrichment analysis, this analysis yielded a total of 1190 DEGs within which included four significant gene modules. In addition, a few hub genes with high degree were found related to the thyroid hormone metabolic process. Our validated experimental results significantly demonstrated two important genes DUOX2 and PDE8B were evaluated in metastatic TC tissues.

DUOX2 was first found in mammalian thyroid gland tissues, mainly in the salivary glands and gastrointestinal tract [23]. DUOX2 activity acts a critical role in the incorporation of thyroglobulin by iodine-bound thyroid peroxidase (TPO). Ginabreda et al. [24] found a significant negative correlation between DUOX2 and TPO in the pathophysiology of TC. However, Lacroix et al. [25] reported that the expression level of DUOX protein was positively correlated with tumor cell differentiation and was more common in TC tissues. Moreover, the promoter of DUOX2 was induced by TSH and insulin in thyroid carcinogenesis [26]. The enrichment results revealed that the DUOX2 gene-related biological processes were activated in the PDMTC group. These evidences enhance the potential role of DUOX2 in the mechanism of metastatic TC.

PDE8B is considered to have the highest affinity for cAMP and regulate cAMP signaling [27]. A recent meta-analysis reported that common genetic variation of PDE8B is significantly related to changes TSH and free T4 [28]. The findings indicated that thyroid hormone levels would be important in epidemiological studies and provided strong evidence that PDE8B is involved in the thyroid TSH signaling pathway [28]. The GSEA analysis results showed that the biological process “regulation of hormone levels (GO: 0010817)” was activated. These evidences indicated that PDE8B may play a key role in regulating the THS levels, which is an independent risk factor for differentiated TC and affects neck lymph node metastasis [29].

Another interesting set of genes including EGR1, TSHR, PAX8, HPN, and TG implicated in our study were associated with cellular hormone-related activities. For example, the thyroid-stimulating hormone receptor (TSHR) which reacts with thyroid-stimulating hormone (also known as “thyrotropin”) is a major regulator of membrane protein and thyroid cell metabolism, including it stimulates the production of thyroxine (T4) and triiodothyronine protamine (T3). Defects in these genes are the cause of many types of hyperthyroidism [30]. Recently, a study demonstrated that TSHR significantly downregulated in well-differentiated TC samples and promoted TC cell invasion and metastasis [31]. Moreover, multivariate analysis showed that TSHR was a critical prognostic factor in predicting metastasis and overall survival [31].

In summary, this study confirms that two new candidate genes, DUOX2 and PDE8B, can be used as prognostic biomarkers or therapeutic targets for patients with metastatic TC. This study will provide important information for elucidating the biological and molecular mechanisms of TC cell metastasis.

## Figures and Tables

**Figure 1:** Box plots of normalized expression data. The grey boxes represent twenty ATC samples, and light blue boxes represent seventeen PDMTC samples. The dash lines in black mean the median of each set of data, which determine the degree of standardization of data through its distribution.

**Figure 2:** Overview of DEGs with clustered heat map, enrichment analysis, and module eigengene results. (a) Clustered heat map of 1190 DEGs. Each row represents a probe, and each column represents a sample. Expression levels are depicted according to the color scale shown at the top. The red color indicated highly expressed mRNAs, and the blue color indicated lowly expressed mRNAs, above or below the median, respectively. (b) GSEA enrichment results of biological processes. The area under the curve represents the distribution of gene expression level, and the color saturation represents the significant level of each biological process. (c) Gene dendrogram and module clustering results. (d) Module eigengenes' correlation matrix with each own coefficient and significant result.

**Figure 3:** Gene coexpression network and enrichment map of significant biological processes. (a) Coexpression network with genes in significant biological processes. The size and color saturation of each node were weighed by the gene expression level and its connections in topological overlap matrix. (b) Enrichment map of significant biological processes. The size and color saturation of each term were defined to interactions among all biological process.

**Figure 4:** Validation of DUOX2 and PDE8B in metastatic TC. (a) The relative gene expression levels of DUOX2 and PDE8B with qRT-PCR method. (b) Immunoblotting analysis results of DUOX2 and PDE8B protein concentration.

**Table 1:** Significant biological processes of GO terminologies.

ID	Description	*P* value	Genes
GO:0042403	Thyroid hormone metabolic process	2.51*E* − 07	DUOX2/DIO1/TPO/HPN/TG/IYD
GO:1901615	Organic hydroxy compound metabolic process	9.04*E* − 07	DUOX2/IL1B/GPER1/MAOA/ACADL/TM7SF2/EPHX2/DIO1/PLCB4/DEGS2/NPC1/LRP2/ACOX2/TPO/HPN/SLC27A2/CITED1/SORD/TG/LDLR/ALDH1A1/IYD
GO:0006590	Thyroid hormone generation	2.12*E* − 06	DUOX2/DIO1/TPO/HPN/IYD
GO:0006575	Cellular modified amino acid metabolic process	3.53*E* − 05	DUOX2/CARNS1/CKMT2/DIO1/TPO/HPN/MTHFD2/ALDH5A1/TG/CKB/IYD
GO:0010817	Regulation of hormone levels	4.87*E* − 05	DUOX2/MME/IL1B/GPER1/PDE8B/EDN3/HSD17B6/INHBA/DIO1/CPE/PTPRN2/HSD17B8/NKX3-1/TPO/HPN/TBX3/TG/ALDH1A1/IYD
GO:0018958	Phenol-containing compound metabolic process	6.60*E* − 05	DUOX2/MAOA/DIO1/TPO/HPN/CITED1/TG/IYD
GO:0042445	Hormone metabolic process	7.92*E* − 05	DUOX2/MME/HSD17B6/DIO1/CPE/HSD17B8/TPO/HPN/TG/ALDH1A1/IYD
GO:0097503	Sialylation	1.95*E* − 04	ST6GAL2/ST6GAL1/ST6GALNAC3/ST3GAL5
GO:0009880	Embryonic pattern specification	2.88*E* − 04	CXXC4/SMAD6/BMP7/CITED1/TBX3/ZBTB16
GO:0042446	Hormone biosynthetic process	3.14*E* − 04	DUOX2/HSD17B6/DIO1/HSD17B8/TPO/TG
GO:0030878	Thyroid gland development	3.35*E* − 04	DUOX2/HHEX/NKX2-1/TG

## Data Availability

The data used to support the findings of this study are available from the corresponding author upon request.

## References

[1] Alvarez J. C., Méndez J. C., Morís C. (2015). *Thyroid Cancer Treatment*.

[2] Yu G. P., Li J. C., Branovan D., McCormick S., Schantz S. P. (2010). Thyroid cancer incidence and survival in the national cancer institute surveillance, epidemiology, and end results race/ethnicity groups. *Thyroid*.

[3] Katikireddi S. V. (2017). Global, regional, and national incidence and prevalence, and years lived with disability for 328 diseases and injuries in 195 countries, 1990-2016: a systematic analysis for the Global Burden of Disease Study 2016. *The Lancet*.

[4] Wang L. Y., Palmer F. L., Nixon I. J. (2014). Multi-organ distant metastases confer worse disease-specific survival in differentiated thyroid cancer. *Thyroid*.

[5] Miller K. D., Siegel R. L., Lin C. C. (2016). Cancer treatment and survivorship statistics, 2016. *CA: A Cancer Journal for Clinicians*.

[6] Shoup M., Stojadinovic A., Nissan A. (2003). Prognostic indicators of outcomes in patients with distant metastases from differentiated thyroid carcinoma. *Journal of the American College of Surgeons*.

[7] Sabra M. M., Ghossein R., Tuttle R. M. (2016). Time course and predictors of structural disease progression in pulmonary metastases arising from follicular cell–derived thyroid cancer. *Thyroid*.

[8] Onda M., Emi M., Yoshida A. (2004). Comprehensive gene expression profiling of anaplastic thyroid cancers with cDNA microarray of 25 344 genes. *Endocrine-Related Cancer*.

[9] Nikiforova M. N., Wald A. I., Roy S., Durso M. B., Nikiforov Y. E. (2013). Targeted next-generation sequencing panel (ThyroSeq) for detection of mutations in thyroid cancer. *The Journal of Clinical Endocrinology & Metabolism*.

[10] Barrett T., Troup D. B., Wilhite S. E. (2011). NCBI GEO: archive for functional genomics data sets—10 years on. *Nucleic Acids Research*.

[11] Landa I., Ibrahimpasic T., Boucai L. (2016). Genomic and transcriptomic hallmarks of poorly differentiated and anaplastic thyroid cancers. *The Journal of Clinical Investigation*.

[12] Herbert J. M. J., Stekel D. J., Mura M., Sychev M., Bicknell R. (2011). *Bioinformatic Methods for Finding Differentially Expressed Genes in cDNA Libraries, Applied to the Identification of Tumour Vascular Targets*.

[13] Camilli G. (1995). The relationship between Fisher’s exact test and Pearson’s chi-square test: a Bayesian perspective. *Psychometrika*.

[14] Zhao H., Cai W., Su S., Zhi D., Lu J., Liu S. (2014). Screening genes crucial for pediatric pilocytic astrocytoma using weighted gene coexpression network analysis combined with methylation data analysis. *Cancer Gene Therapy*.

[15] Zhang B., Horvath S. (2005). A general framework for weighted gene co-expression network analysis. *Statistical Applications in Genetics & Molecular Biology*.

[16] Langfelder P., Horvath S. (2007). Eigengene networks for studying the relationships between co-expression modules. *BMC Systems Biology*.

[17] Kanehisa G. (2000). KEGG: kyoto encyclopedia of genes and genomes [J]. *Nucleic Acids Research*.

[18] Yu G., Wang L. G., Han Y., He Q. Y. (2012). clusterProfiler: an R package for comparing biological themes among gene clusters. *OMICS: A Journal of Integrative Biology*.

[19] Subramanian A., Tamayo P., Mootha V. K. (2005). Gene set enrichment analysis: a knowledge-based approach for interpreting genome-wide expression profiles. *Proceedings of the National Academy of Sciences of the United States of America*.

[20] Hannallah J., Rose J., Guerrero M. A. (2013). Comprehensive literature review: recent advances in diagnosing and managing patients with poorly differentiated thyroid carcinoma. *International Journal of Endocrinology*.

[21] Lote H., Bhosle J., Thway K., Newbold K., O'Brien M. (2014). Epidermal growth factor mutation as a diagnostic and therapeutic target in metastatic poorly differentiated thyroid carcinoma: a case report and review of the literature. *Case Reports in Oncology*.

[22] Langfelder P., Mischel P. S., Horvath S. (2013). When is hub gene selection better than standard meta-analysis?. *PLoS One*.

[23] Geiszt M., Witta J., Baff J., Lekstrom K., Leto T. L. (2003). Dual oxidases represent novel hydrogen peroxide sources supporting mucosal surface host defense. *FASEB Journal*.

[24] Ginabreda M. G., Cardoso L. C., Nobrega F. M. (2008). Negative correlation between thyroperoxidase and dual oxidase H_2_O_2_-generating activities in thyroid nodular lesions. *European Journal of Endocrinology*.

[25] Lacroix L., Nocera M., Mian C. (2001). Expression of nicotinamide adenine dinucleotide phosphate oxidase flavoprotein DUOX genes and proteins in human papillary and follicular thyroid carcinomas. *Thyroid*.

[26] Cardoso-Weide L. C., Cardoso-Penha R. C., Costa M. W., Ferreira A. C. F., Carvalho D. P., Santisteban P. S. (2015). DuOx2 promoter regulation by hormones, transcriptional factors and the coactivator TAZ. *European Thyroid Journal*.

[27] Bender A. T., Beavo J. A. (2006). Cyclic nucleotide phosphodiesterases: molecular regulation to clinical use. *Pharmacological Reviews*.

[28] Taylor P. N., Panicker V., Sayers A. (2011). A meta-analysis of the associations between common variation in the PDE8B gene and thyroid hormone parameters, including assessment of longitudinal stability of associations over time and effect of thyroid hormone replacement. *European Journal of Endocrinology*.

[29] McLeod D. S., Cooper D. S., Ladenson P. W. (2014). Prognosis of differentiated thyroid cancer in relation to serum thyrotropin and thyroglobulin antibody status at time of diagnosis. *Thyroid*.

[30] Yuan Z. F., Mao H. Q., Luo Y. F., Wu Y. D., Shen Z., Zhao Z. Y. (2008). Thyrotropin receptor and thyroid transcription factor-1 genes variant in Chinese children with congenital hypothyroidism. *Endocrine Journal*.

[31] Liu T., Men Q., Su X. (2017). Downregulated expression of TSHR is associated with distant metastasis in thyroid cancer [J]. *Oncology Letters*.

